# High-Density Lipoprotein Cholesterol in Young Nondiabetic Coronary Heart Disease Patients

This article has been retracted.

**DOI:** 10.1155/2021/2970568

**Published:** 2021-07-13

**Authors:** Ziyang Hu, Jingle Cui, Xueshan Li, Yaohui Zhou, Lu Cai, Shibin Zhang

**Affiliations:** ^1^Department of Cardiology, Zhongshan Hospital of Traditional Chinese Medicine, Zhongshan 528400, China; ^2^Department of Cardiothoracic Surgery, Zhongshan Hospital of Traditional Chinese Medicine, Zhongshan 528400, China; ^3^Emergency Department, Zhongshan Hospital of Traditional Chinese Medicine, Zhongshan 528400, China; ^4^Department of Clinical Laboratory, Zhongshan Hospital of Traditional Chinese Medicine, Zhongshan 528400, China; ^5^Graduate School of Hunan University of Chinese Medicine, Changsha 410208, China

## Abstract

**Objective:**

To investigate the association between the lipid profiles and coronary heart disease (CHD) in nondiabetic patients younger than 65 years of age.

**Method:**

424 patients were enrolled in this study from January 2019 to December 2020. All the patients were screened for clinically indicated coronary angiography. They were divided into two groups according to the coronary angiography results: 340 patients with the presence of CHD (at least one coronary artery stenosis ≥50%) were classified as the CHD group, and the rest with the absence of CHD comprised the normal group. The demographic data and lipid profiles were compared.

**Result:**

CHD was higher in males than females (84.5% *vs*. 62.2%, *P* < 0.001). In the CHD group, the level of high‐density lipoprotein cholesterol (HDL-C) was lower (*P* < 0.001), while the triglyceride (TG)/HDL-C ratio was higher (*P*=0.022). No significant differences were shown between the two groups in terms of age, family history of CHD, hypertension, and the levels of TC, TG, and LDL-C. Gender differences were further explored. In men, except for the level of HDL-C which was significantly lower in the CHD group than that in the normal group (*P*=0.017), parameters were comparable. A binary logistic regression model further indicated that HDL-C was associated with CHD (OR = 0.137, 95%CI: 0.031–0.594, *P*=0.008). Also, with the increase of the number of coronary artery with lesions, the levels of HDL-C decreased significantly in men. In women, no differences were observed between the CHD group and normal group.

**Conclusion:**

HDL-C may be inversely associated with the risk of CHD in young nondiabetes patients, especially in men. More research is needed to confirm it.

## 1. Introduction

In spite of a remarkable decline in death rates from cardiovascular disease (CVD) observed over the last decades, CVD still remains the leading cause of total years of life lost globally [1, 2]. Coronary heart disease (CHD) and stroke were the most common causes of CVD deaths. The pathological basis for CHD and stroke was atherosclerosis featured by the accumulation of plaques in vessel walls [3]. Dyslipidemia is an important risk factor for CHD and stroke. A strong relationship has been established between a higher level of low-density lipoprotein cholesterol (LDL-C) or a lower level of high-density lipoprotein cholesterol (HDL-C) with an increasing risk for CHD [4]. Moreover, an increasing amount of evidence has showed that an elevated level of triglyceride (TG) is independently associated with an increased risk of CHD [4, 5]. Recently, the ratio of TG/HDL-C was found to be closely related to insulin resistance, metabolic syndrome, and diabetes [6–9]. Known as a well-defined atherogenic plasma index, the TG/HDL-C ratio was also indicated to be an important predictor for CHD [10–12] by reflecting the balance between atherogenic and protective lipoproteins [13].

Gender differences have also been reported in the prevalence, clinical presentation, and outcomes of CVD [14, 15]. Due to the higher life expectancy than men do, women form a larger proportion of the elderly population in which the prevalence of CVD is the highest. However, when adjusted for differences in age distribution, the CVD mortality and morbidity rates are the highest in men than that in women. So far, the basic epidemiological characteristics of CHD are diseases of the middle-aged and elderly population, but there is a pronounced tendency of younger age [16]. However, studies regarding the relation between CHD and lipid profiles according to gender have been rarely reported, especially in those young adults.

Thus, in the present study, we conducted a retrospective study to investigate the association between the lipid profiles and CHD in nondiabetic patients younger than 65 years of age.

## 2. Methods

### 2.1. Patients

424 patients admitted to the Zhongshan Hospital of Traditional Chinese Medicine from January 2019 to December 2020 were enrolled in this study. All the patients were screened for clinically indicated coronary angiography. The exclusion criteria were as follows: (1) younger than 18 or older than 65; (2) diagnosed as diabetes; (3) severe congenital heart disease; (4) severe valvular heart disease; (5) high-powered heart disease, such as hyperthyroidism and severe anemia; (6) pulmonary heart disease; (7) hypertrophic obstructive cardiomyopathy; (8) severe liver and/or renal insufficiency and malignancy; or (9) severe hematologic disorders. The patients were divided into two groups according to the coronary angiography results: 340 patients with the presence of CHD (at least one coronary artery stenosis ≥50%) were classified as the CHD group, and the rest with the absence of CHD comprised the normal group. The study protocol was approved by the institutional ethics committee of Zhongshan Hospital of Traditional Chinese Medicine, and informed consent for their clinical data to be used for research purposes was obtained from all participants.

### 2.2. Data Collection

The demographic data and laboratory data were obtained from case records. The demographic data included age, gender, body mass index (BMI), family history of CHD, hypertension, diabetes, and smoking. Hypertension was defined as a repeated systolic blood pressure of ≥140 mmHg and/or diastolic blood pressure of ≥90 mmHg (at least 2 times in different environments) or currently taking antihypertensive drugs. Diabetes was defined as fasting plasma glucose ≥7.0 mmol/L; 2-hour plasma glucose >11.1 mmol/L during an oral glucose tolerance test (OGTT); or active use of hypoglycemic drugs. Smoking was determined as a previous history of smoking or active smoking. The laboratory data included lipid profiles, cardiac markers, biochemical parameters, and hemogram. Some parameters were obtained during admission to the hospital. After an overnight fasting, blood samples for lipid profiles, including total cholesterol (TC), TG, HDL-C, and LDL-C, were obtained. All the blood samples were delivered into the laboratory of the hospital. The blood samples for lipid profiles were analyzed using standard methods, without any delay.

### 2.3. Coronary Angiography

Coronary angiography was performed using the UNIQ Clarify FD20 equipment (Philips, the Netherlands). All procedures followed the standard American College of Cardiology (ACC)/American Heart Association (AHA) guidelines for coronary angiography. The coronary angiograms were evaluated by experienced interventional cardiologists.

### 2.4. Statistical Analysis

Continuous variables were presented as the mean ± standard error (SD), and categorical variables were presented as frequencies and percentages. Appropriate statistical tests were used for comparison, including the Mann–Whitney *U* test, chi-square test, Fisher's exact test, and one-way ANOVA. A binary logistic regression model was used to investigate the risk factors of CHD in nondiabetic patients. The presence or absence of CHD was used as a dependent variable. The variables demonstrating differences between patients with or without CHD (entry criterion *P* < 0.1) or those that had been reported to be associated with CHD were included in the regression analysis with the enter method. The statistical analysis was performed with the Statistical Package for Social Sciences (SPSS, version 16.0 for Windows). *P* < 0.05 was considered statistically significant.

## 3. Results

The average age of 424 patients was 53.1 ± 8.5 (years) (range: 23–65).  Table 1 showed the baseline characteristics of the patients. CHD was higher in males than females (84.5% *vs*. 62.2%, *P* < 0.001). More smokers were in the CHD group than that in the normal group (*P*=0.001). In the CHD group, the TG/HDL-C ratio was higher (*P*=0.022), while the levels of HDL-C were lower (*P* < 0.001). No significant differences were shown between the two groups in terms of age, family history of CHD, hypertension, and the levels of TC and LDL-C.

Gender differences were further investigated. In men, except for the level of HDL-C which was significantly lower in the CHD group than that in the normal group (*P*=0.017), parameters were comparable between these two groups (Table 2). However, in women, no significant differences were observed between the CHD group and normal group (Table 2). The binary logistic regression model indicated that, in nondiabetic men, HDL-C was associated with CHD (OR = 0.137, 95%CI: 0.031–0.594, *P*=0.008), but showed no associations with the remaining risk factors including hypertension, smoking, family history of CHD, TC, TG, LDL-C, and TG/HDL-C.

Figure 1 presents the levels of HDL-C grouped by the number of coronary artery with lesions in nondiabetic men. The average levels of HDL-C in each group were 1.16 ± 0.42 (mmol/L, normal group, *n* = 53), 1.03 ± 0.24 (mmol/L, single-vessel group, *n* = 87), 1.02 ± 0.25 (mmol/L, two-vessel group, *n* = 93), and 0.99 ± 0.24 (mmol/L, three-vessel group, *n* = 109), respectively. A significant decrease was observed among these groups (*P*=0.044). Further multiple comparisons showed that the level of HDL-C was significant lower in the three-vessel group than in the normal group (*P*=0.037).

## 4. Discussion

CHD is one of the leading causes of death worldwide with a trend to be younger, despite the remarkable progress in the research of molecular and pathological mechanisms and treatment of it [17–23]. Identifying risk factors and adequate management is one of the corner stones of preventing CHD. It is meaningful to explore the risk factors of CHD in young adults. Diabetes is associated with increased CHD morbidity and mortality. Patients with diabetes are also more prone to heart failure, arrhythmias, and sudden cardiac death. Furthermore, coronary interventions performed in such high-risk patients have worse outcomes. “Atherogenic dyslipidaemia” is a characteristic of lipid profiles in type 2 diabetes mellitus [24]. Thus, in order to eliminate the interference of diabetes on results, we conducted this retrospective study in nondiabetic patients younger than 65 years of age. The results of the present study indicated that the levels of HDL-C and TG/HDL-C ratio might be associated with the risk of CHD in nondiabetic patients younger than 65 as well. However, the level of LDL-C between the CHD group and normal group showed no significant differences. We speculated that it might be related to the age- and gender- specific differences. It has been reported that fluctuating increasing and decreasing LDL-C levels occurred with phases of aging in both sexes [25].

HDL-C lipoproteins are the smallest (5–17 nm) and densest (1.063–1.210 kg/L) in the plasma. Many clinical and epidemiological studies have clearly demonstrated that the HDL-C is inversely correlated with the risk of CHD and is a critical and independent component of predicting this risk [26]. Our results confirmed this opinion again in young nondiabetic patients. The mechanisms that HDL-C is associated with CHD are currently unclear. HDL-C is demonstrated to play antioxidative and anti-inflammatory effects as well as improvement of endothelial function, alongside the prominent role in reverse cholesterol transport [27–29]. In addition, HDL-C can have antithrombotic and profibrinolytic effects [30]. Thus, the lower level of HDL-C might weaken these protective effects, which lead to the occurrence of atherosclerosis, the most common cause of CAD pathogenesis.

Recently, the TG/HDL-C ratio was also reported to be related to CHD. It has been demonstrated that the TG/HDL-C ratio may be an important predictor for an acute coronary syndrome in the young adult population and can even be used to prevent myocardial infarction in young adults [31]. In the present study, the TG/HDL-C ratio was also significantly higher in young nondiabetic patients with CHD when compared to those without CHD.

Gender differences proved to exist in the development of CHD. Male gender was known to have a greater risk of developing CVD than women due to the protective effect of hormones, as long as women are of childbearing age. As shown in our study, 85.0% of CHD patients were men. Whether there were gender differences of lipid profiles in CHD is still rarely reported, especially in those young adults. The results of the present study indicated that in those nondiabetic men younger than 65 years of age, the level of HDL-C might be associated with the risk of CHD, and with the decline of the level of HDL-C, the severity of coronary artery disease increased. However, the TG/HDL-C ratio showed no significant differences even though it was higher in the CHD group. We deemed that this might be related to the small sample size. In addition, all the lipid parameters were comparable between the CHD group and normal group in women. These might be due to the protective effect of hormones. Sample size should be also considered. More data are needed to confirm it.

## 5. Conclusions

Dyslipidemia is one of the most recognized risk factors associated with CHD, and many lipid parameters were demonstrated related to the occurrence of CHD; however, they may fall short when determining the definite cardiovascular risk in young adults. Our study suggests that HDL-C may be inversely associated with the risk of CHD in young nondiabetes CHD patients, especially in men. More research is needed to confirm it.

## Figures and Tables

**Figure 1:** The levels of HDL-C in nondiabetic men grouped by different numbers of coronary artery with lesion (*P* < 0.05) (one-way ANOVA was used for the analysis, and ^∗^ denotes further multiple comparisons: normal *vs*. three vessels (*P* < 0.05)).

**Table 1:** Characteristics of patients without diabetes in the CHD group and normal group.

	CHD group (*n* = 340)	Normal group (*n* = 84)	*P* value
Age (y)^a^	53.2 ± 8.2	52.8 ± 9.6	0.929
Gender^b^			<0.001^*∗*^
Female	51 (62.2)	31 (37.8)	
Male	289 (84.5)	53 (15.5)	
Family history of CHD, *n* (%)^b^	30 (8.8)	7 (8.3)	0.887
Hypertension, *n* (%)^b^	182 (53.5)	38 (45.2)	0.173
Smoking, *n* (%)^b^	164 (48.2)	23 (27.4)	0.001^*∗*^
Lipid profiles^a^			
TC (mmol/l)	5.12 ± 1.43	5.06 ± 1.16	0.842
TG (mmol/l)	1.88 ± 1.42	1.79 ± 1.42	0.261
HDL-C (mmol/l)	1.04 ± 0.26	1.21 ± 0.39	<0.001^*∗*^
LDL-C (mmol/l)	3.11 ± 1.17	2.97 ± 0.89	0.418
TG/HDL-C ratio	1.99 ± 1.80	1.71 ± 1.61	0.022^*∗*^

^a^Mann–Whitney *U* test was used for the analysis. ^b^Chi-square test was used for the analysis. ^*∗*^A statistically significant difference (*P* < 0.05).

**Table 2:** Characteristics of patients without diabetes in the CHD group and normal group in different genders.

	Male gender			Female gender		
	CHD group	Normal group	*P* value	CHD group	Normal group	*P* value
*n*	289	53		51	31	
Age (y)^a^	52.6 ± 8.5	50.7 ± 10.1	0.314	56.5 ± 6.1	56.4 ± 7.7	0.935
Family history of CHD, *n* (%)	29 (10.0)	6 (11.3)	0.776^b^	1 (2.0)	1 (3.2)	1.000^c^
Hypertension, *n* (%)^b^	149 (51.6)	21 (39.6)	0.110	33 (64.7)	17 (54.8)	0.374
Smoking, *n* (%)	162 (56.1)	22 (41.5)	0.051^b^	2 (3.9)	1 (3.2)	1.000^c^
Lipid profiles^a^						
TC (mmol/l)	5.06 ± 1.42	4.84 ± 1.12	0.304	5.44 ± 1.49	5.42 ± 1.14	0.841
TG (mmol/l)	1.86 ± 1.43	1.73 ± 1.30	0.238	1.99 ± 1.33	1.88 ± 1.62	0.351
HDL-C (mmol/l)	1.01 ± 0.24	1.16 ± 0.42	0.017^*∗*^	1.22 ± 0.28	1.28 ± 0.33	0.332
LDL-C (mmol/l)	3.11 ± 1.16	2.88 ± 0.88	0.199	3.08 ± 1.26	3.11 ± 0.89	0.752
TG/HDL-C	2.02 ± 1.84	1.72 ± 1.52	0.094	1.85 ± 1.56	1.68 ± 1.80	0.320

^a^Mann–Whitney *U* test was used for the analysis. ^b^Chi-square test was used for the analysis. ^c^Fisher's exact test was used for the analysis. ^*∗*^A statistically significant difference (*P* < 0.05).

## Data Availability

The data used to support the findings of this study are available from the corresponding author upon request.

## References

[1] (2017). Global, regional, and national age-sex specific mortality for 264 causes of death, 1980–2016: a systematic analysis for the Global burden of disease study 2016. *The Lancet*.

[2] Virani S. S., Alonso A., Aparicio H. J. (2021). Heart disease and stroke statistics-2021 update: a report from the American heart association. *Circulation*.

[3] Tao J., Qiu J., Lu L. (2021). ZBTB20 positively regulates oxidative stress, mitochondrial fission, and inflammatory responses of ox-LDL-induced macrophages in atherosclerosis. *Oxidative Medicine and Cellular Longevity*.

[4] Reiner Ž. (2017). Hypertriglyceridaemia and risk of coronary artery disease. *Nature Reviews Cardiology*.

[5] Peng J., Luo F., Ruan G., Peng R., Li X. (2017). Hypertriglyceridemia and atherosclerosis. *Lipids in Health and Disease*.

[6] Lin D., Qi Y., Huang C. (2018). Associations of lipid parameters with insulin resistance and diabetes: a population-based study. *Clinical Nutrition*.

[7] Gasevic D., Frohlich J., Mancini G. J., Lear S. A. (2014). Clinical usefulness of lipid ratios to identify men and women with metabolic syndrome: a cross-sectional study. *Lipids in Health and Disease*.

[8] Zhou M., Zhu L., Cui X. (2016). The triglyceride to high-density lipoprotein cholesterol (TG/HDL-C) ratio as a predictor of insulin resistance but not of *β* cell function in a Chinese population with different glucose tolerance status. *Lipids in Health and Disease*.

[9] Chen Z., Hu H., Chen M. (2020). Association of triglyceride to high-density lipoprotein cholesterol ratio and incident of diabetes mellitus: a secondary retrospective analysis based on a Chinese cohort study. *Lipids in Health and Disease*.

[10] Gaziano J. M., Hennekens C. H., O’Donnell C. J., Breslow J. L., Buring J. E. (1997). Fasting triglycerides, high-density lipoprotein, and risk of myocardial infarction. *Circulation*.

[11] Zhou L., Mai J., Li Y. (2020). Triglyceride to high-density lipoprotein cholesterol ratio and risk of atherosclerotic cardiovascular disease in a Chinese population. *Nutrition, Metabolism and Cardiovascular Diseases*.

[12] Dai X.-Y., Zheng Y.-Y., Tang J.-N. (2019). Triglyceride to high-density lipoprotein cholesterol ratio as a predictor of long-term mortality in patients with coronary artery disease after undergoing percutaneous coronary intervention: a retrospective cohort study. *Lipids in Health and Disease*.

[13] Millan J., Pinto X., Munoz A. (2009). Lipoprotein ratios: physiological significance and clinical usefulness in cardiovascular prevention. *Vascular Health and Risk Management*.

[14] Kuznetsova T. (2018). Sex differences in epidemiology of cardiac and vascular disease. *Advances in Experimental Medicine and Biology*.

[15] Khamis R. Y., Ammari T., Mikhail G. W. (2016). Gender differences in coronary heart disease. *Heart*.

[16] Masic I., Rahimic M., Dilic M., Kadribasic R., Toromanovic S. (2011). Socio-medical characteristics of coronary disease in Bosnia and Herzegovina and the world. *Materia Socio Medica*.

[17] Jusic A., Devaux Y., Devaux Y. (2020). Mitochondrial noncoding RNA-regulatory network in cardiovascular disease. *Basic Research in Cardiology*.

[18] Wang J., Zhou H. (2020). Mitochondrial quality control mechanisms as molecular targets in cardiac ischemia-reperfusion injury. *Acta Pharmaceutica Sinica B*.

[19] Lobo-Gonzalez M., Galán-Arriola C., Rossello X. (2020). Metoprolol blunts the time-dependent progression of infarct size. *Basic Research in Cardiology*.

[20] Zhou H., Wang S., Zhu P., Hu S., Chen Y., Ren J. (2018). Empagliflozin rescues diabetic myocardial microvascular injury via AMPK-mediated inhibition of mitochondrial fission. *Redox Biology*.

[21] Heusch G. (2019). Coronary microvascular obstruction: the new frontier in cardioprotection. *Basic Research in Cardiology*.

[22] Kleinbongard P. (2020). Cardioprotection by early metoprolol- attenuation of ischemic vs. reperfusion injury?. *Basic Research in Cardiology*.

[23] Tao J., Wang Y., Li L., Zheng J., Liang S. (2020). Critical roles of ELVOL4 and IL-33 in the progression of obesity-related cardiomyopathy via integrated bioinformatics analysis. *Frontiers in Physiology*.

[24] Katsiki N., Tentolouris N., Mikhailidis D. P. (2017). Dyslipidaemia in type 2 diabetes mellitus. *Current Opinion in Cardiology*.

[25] Zhang P., Su Q., Ye X. (2020). Trends in LDL-C and non-HDL-C levels with age. *Aging and Disease*.

[26] Wang H. H., Garruti G., Liu M., Portincasa P., Wang D. Q.-H. (2017). Cholesterol and lipoprotein metabolism and atherosclerosis: recent advances in reverse cholesterol transport. *Annals of Hepatology*.

[27] Annema W., von Eckardstein A. (2013). High-density lipoproteins. *Circulation Journal*.

[28] Lüscher T. F., Landmesser U., von Eckardstein A., Fogelman A. M. (2014). High-density lipoprotein. *Circulation Research*.

[29] Besler C., Heinrich K., Riwanto M., Luscher T., Landmesser U. (2010). High-density lipoprotein-mediated anti-atherosclerotic and endothelial-protective effects: a potential novel therapeutic target in cardiovascular disease. *Current Pharmaceutical Design*.

[30] Griffin J. H., Kojima K., Banka C. L., Curtiss L. K., Fernández J. A. (1999). High-density lipoprotein enhancement of anticoagulant activities of plasma protein S and activated protein C. *Journal of Clinical Investigation*.

[31] Dogan C., Bayram Z., Karagoz A. (2019). Is elevated triglyceride high density lipoprotein cholesterol ratio a risk factor that causes acute coronary syndrome to appear earlier?. *Bratislava Medical Journal*.

